# Evaluation of Prophylactic and Therapeutic Effects of Tramadol and Tramadol Plus Magnesium Sulfate in an Acute Inflammatory Model of Pain and Edema in Rats

**DOI:** 10.3389/fphar.2018.01326

**Published:** 2018-11-16

**Authors:** Dragana Srebro, Sonja Vučković, Aleksandar Milovanović, Katarina Savić Vujović, Milica Prostran

**Affiliations:** ^1^Department of Pharmacology, Clinical Pharmacology and Toxicology, Faculty of Medicine, University of Belgrade, Belgrade, Serbia; ^2^Institute of Occupational Health Dr Dragomir Karajovic, Faculty of Medicine, University of Belgrade, Belgrade, Serbia

**Keywords:** tramadol, magnesium sulfate, preemptive therapy, emptive therapy, drug interaction, antihyperalgesic effect

## Abstract

**Background:** Inflammatory pain is the most commonly treated clinical pain, since it develops following trauma or surgery, and accompanies rheumatic or arthritic diseases. Tramadol is one of the most frequently used opioid analgesics in acute and chronic pain of different origin. Magnesium is a widely used dietary supplement that was recently shown to be a safe analgesic drug in different models of inflammatory pain.

**Aim:** This study aimed to evaluate the effects of systemically or locally injected tramadol with/without systemically injected magnesium sulfate in prophylactic or therapeutic protocols of application in a rat model of somatic inflammation.

**Methods:** Inflammation of the rat hind paw was induced by an intraplantar injection of carrageenan (0.1 ml, 0.5%). The antihyperalgesic/antiedematous effects of tramadol (intraperitoneally or intraplantarly injected), and tramadol-magnesium sulfate (subcutaneously injected) combinations were assessed by measuring the changes in paw withdrawal thresholds or paw volume induced by carrageenan. The drugs were administered before or after inflammation induction.

**Results:** Systemically administered tramadol (1.25–10 mg/kg) before or after induction of inflammation reduced mechanical hyperalgesia and edema with a maximal antihyperalgesic/antiedematous effect of about 40–100%. Locally applied tramadol (0.125 mg/paw) better reduced edema (50–100%) than pain (20–50%) during 24 h. Administration of a fixed dose of tramadol (1.25 mg/kg) with different doses of magnesium led to a dose-dependent enhancement and prolongation of the analgesic effect of tramadol both in prevention and treatment of inflammatory pain. Magnesium increases the antiedematous effect of tramadol in the prevention of inflammatory edema while reducing it in treatment.

**Conclusion:** According to results obtained in this animal model, systemic administration of low doses of tramadol and magnesium sulfate given in combination is a potent, effective and relatively safe therapeutic option for prevention and especially therapy of somatic inflammatory pain. The best result is achieved when tramadol is combined with magnesium sulfate at a dose that is equivalent to the average human recommended daily dose and when the drugs are administered when inflammation is maximally developed.

## Introduction

Inflammatory pain and edema can be caused by different clinical conditions in which inflammation is triggered by tissue injury, heat, an inadequate immune response and infection. Inflammatory pain that is very intense and/or long-lasting can lead to the development of chronic pain. In Europe, about 20% of the adult population has moderate to severe non-cancer chronic pain in the course of 1 month (Reid et al., 2011). Conditions following inflammatory pain can be difficult to treat using a one-drug therapy, since this pain includes various mechanisms of nociceptive modulation and transmission, and also inflammation can worse pain sensitivity (Libby, 2007).

Non-steroidal anti-inflammatory drugs (NSAIDs), given by oral or topical route, are the main and effective drugs for therapy of inflammatory pain. However, their oral use is limited by side effects and insufficient efficacy against severe pain (Grosser et al., 2018). Opioid analgesics may be used for severe inflammatory pain, however their use, especially longer term, is limited due to increased risk of side effects, tolerance, and dependence (Yaksh and Wallace, 2018). Thus, there is a clinical need for a novel strategy to treat inflammatory pain.

Tramadol is an atypical and centrally-acting opioid analgesic. Its analgesic effect is achieved by week activation of mu-opioid receptors, but also through inhibition of the re-uptake of both serotonin and noradrenaline (Grond and Sablotzki, 2004). Tramadol is effective in both acute and chronic pain states; it relieves pain induced by trauma, renal or biliary colic, and cancer-related pain. Compared to strong opioids, tramadol has an upper limit of efficacy, but also produces less respiratory depression, dependence and constipation.

Magnesium is a trace element that acts as a cofactor of enzymes, as a regulator of transmembrane ion fluxes by pumps, carriers and channels, and as a regulator of neurotransmitter (e.g., acetylcholine, norepinephrine) release, participating in metabolic processes, protein synthesis, vasodilatation and neuromuscular excitability (Shimosawa et al., 2004; Guiet-Bara et al., 2007). Our previous results showed that magnesium as a single drug in a single dose of magnesium sulfate has analgesic effect in somatic and visceral inflammatory pain (Srebro et al., 2014a, Vuckovic et al., 2015; Srebro et al., 2018a). The analgesic effect is produced after systemic, but not after local peripheral administration (Srebro et al., 2014a). Magnesium reduces inflammatory pain as both a prophylactic and therapeutic drug (Srebro et al., 2014a). The analgesic effect of magnesium in inflammatory pain is achieved by modulating nitric oxide synthesis (Srebro et al., 2014a, Vuckovic et al., 2015; Srebro et al., 2016a). In the general population, magnesium is a widely used dietary supplement, and it could potentially interact with other drugs, such as antibiotics (Adepoju-Bello et al., 2008).

The objective of the present study was to investigate the possible antihyperalgesic and antiedematous effect of tramadol alone and in combination with magnesium sulfate after systemic and local peripheral administration, in the prevention and treatment of inflammatory pain and edema, using a suitable animal model and different protocols for use of the drugs.

## Materials and Methods

### Animals

Adult male Wistar rats (220–260 g) were used in the experiments. Animals were housed three per Plexiglas cage (42.5 × 27 × 19 cm) under standard laboratory conditions of temperature (22 ± 1°C), relative humidity (60%), and a 12 h light/dark cycle, with lights on at 08:00 h. Food and water were freely available, except during the experimental procedures. The animals were fed with standard rat pellets. Rats were habituated to the laboratory environment for at least 2 h before the experiments. All experimental groups were comprised of 6 rats. The experiments were conducted by the same experimenter on consecutive days to avoid diurnal variations in the behavioral tests. Each animal was used only once, it received only one dose of the tested drug and was killed at the end of the experiments by an intraperitoneal injection of sodium thiopental (200 mg/kg). The experiments were approved by the Local Ethical Committee of the Medical University (permit No. 4946/2) and the Ethical Council of the Ministry of Agriculture, Forestry and Water Management, which are in compliance with the European Community Council Directive of November 24th, 1986 (86/609/EEC) and the International Association for the Study of Pain (IASP) Guidelines for the Use of Animals in Research.

### Administration of Drugs

Magnesium sulfate (Magnesio Solfato; S.A.L.F. Spa-Cenate Sotto, Bergamo, Italy), tramadol hydrochloride (Trodon, solution for injection, Hemofarm AD, Vršac, Serbia) and λ-carrageenan (Sigma-Aldrich, St. Louis, MO, United States) were dissolved in 0.9% NaCl and injected subcutaneously (s.c.) or intraperitoneally (i.p.) at a final volume of 2 ml/kg, and intraplantarly (i.pl.) at a final volume of 0.1 ml *per* paw. To test whether the 0.9% NaCl injection had any effect on the nociception, the same volume of 0.9% NaCl was administered to a control group of rats.

### Carrageenan Model of Acute Local Inflammation

The i.pl. injection of 100 μl 0.5% λ-carrageenan in the right hind paw was used to induce unilateral hind paw inflammation in the rat (Srebro et al., 2014a). The injection of carrageenan produces more persistent pain/hyperalgesia and edema which the animals cannot control. These tests evaluate both peripheral (nociceptive afferent fibers) and central mechanisms and both neurogenic and non-neurogenic inflammatory responses of hyperalgesia and edema.

### Measurement of the Hyperalgesia by von Frey’s Electronic Pressure-Meter Test

The carrageenan-induced pain test assesses the spinal response to pain by measuring the paw withdrawal reflex threshold following exposure to a mechanical stimulus. We conducted the test as previously described in detail (Srebro et al., 2014a,b). In brief, the von Frey filament was applied to the plantar surface of the tested paw until the paw withdrawal threshold occurred. The intensity of the stimulus (in grams) was automatically record and displayed on the von Frey apparatus (electronic von Frey Anesthesiometer, Model 2390, IITC Life Science, Woodland Hills, CA, United States). Measurements were performed four times in each rat, and the average of the middle three values calculated. The hind paw withdrawal threshold to mechanical stimuli was measured at 0, 1, 2, 3, 4, 5, 6, and 24 h after an i.pl. injection of carrageenan. Animals displaying a baseline paw withdrawal threshold of more than 65 g were excluded from the study.

### Measurement of the Edema by Plethysmometer Test

The carrageenan-induced inflammatory edema on the rat hind paw was measured by immersing the paw up to tibiotarsal joint in the cylinder of the apparatus (Plethysmometer, Model Almemo 2390-5, IITC Life Science, Woodland Hills, CA, United States), as we previously described in detail (Srebro et al., 2018b). The paw volume (in ml) was measured after measurements of hyperalgesia test in each time points.

### Data Analysis

The intensity of the hyperalgesia/edema was quantified as the difference in pressures [d (g)] applied/difference in paw volume [d (ml)] before and after injection of carrageenan (control d), or before and after injection of carrageenan plus the drugs (test d) (Srebro et al., 2014a,b, 2018b).

Agents capable of reducing the d(g) were recognized as possessing antihyperalgesic activity. The analgesic activity (AA %) for each rat was calculated according to the formula (Srebro et al., 2014a,b):

$$\begin{array}{c} \%\mathrm{AA}=[(\mathrm{control}\;\mathrm{group}\;\mathrm{average}\;d(g)-\mathrm{test}\;\mathrm{group}\;\mathrm{average}\;d(g)\\ \mathrm{of}\;\mathrm{each}\;\mathrm{rat})/(\mathrm{control}\;\mathrm{group}\;\mathrm{average}\;d(g))]\;\times 100. \end{array}$$

A reducing of the difference in volume (dv) was designated as antiedematous activity (AE%) and was calculated for each rat in one group using the following formula (Srebro et al., 2018b):

$$\begin{array}{c} \%\mathrm{AE}=[(\mathrm{the}\;\mathrm{average}\;\mathrm{dv}\;\mathrm{in}\;\mathrm{the}\;\mathrm{control}\;\mathrm{group}-\mathrm{the}\;\mathrm{average}\\ \mathrm{dv}\;\mathrm{observed}\;\mathrm{in}\;\mathrm{each}\;\mathrm{rat}\;\mathrm{in}\;\mathrm{the}\;\mathrm{tested}\;\mathrm{group})/\\ \mathrm{the}\;\mathrm{average}\;\mathrm{dv}\;\mathrm{in}\;\mathrm{the}\;\mathrm{control}\;\mathrm{group})]\times 100. \end{array}$$

The time-course of the antihyperalgesic/antiedematous responses to the individual drugs and their combinations were defined as the first and last time points, when a statistically significant difference in the paw withdrawal threshold/paw volume between the treated and control groups exists.

### Study Design

The tested drugs were evaluated after systemic and local peripheral administrations in prophylactic and therapeutic protocols of use (Table 1).

**Table 1:** Experimental protocol.

Time	-10 min	-5 min	0 min	1 h	1 h 55 min	2 h	3–6 h 24 h
							
Predrug measurments	Inj.	Inj.	Inj.	Postdrug measurments	Inj.	Inj.	Postdrug measurments
	NaCl i.p.		NaCl i.pl.				
	NaCl i.p.		Carr i.pl.				
	T i.p.		Carr i.pl.				
			Carr i.pl.		NaCl i.p.		
			Carr i.pl.		T i.p.		
			NaCl CL +Carr i.pl.				
			NaCl T CL +Carr i.pl.				
			T IL +Carr i.pl.				
		NaCl s.c.	Carr i.pl.				
		Mg s.c.	Carr i.pl.				
			Carr i.pl.		NaCl s.c.		
			Carr i.pl.			Mg s.c.	
	NaCl i.p.	NaCl s.c.	Carr i.pl.				
	T i.p.	Mg s.c.	Carr i.pl.				
			Carr i.pl.		NaCl i.p.	NaCl s.c.	
			Carr i.pl.		T i.p.	Mg s.c.	


*The effects of tramadol, magnesium sulfate, and combinations of tramadol and magnesium sulfate on paw withdrawal threshold and paw volume in rats were evaluated. The control animals received the corresponding injections of 0.9% NaCl (NaCl) instead of test compounds. i.p., intraperitoneal; s.c., subcutaneous; i.pl., intraplantar; inj., injection; IL, ipsilateral; CL, contralateral; Carr, carrageenan; Mg, magnesium sulfate; T, tramadol.*

Three distinct schemes of prophylactic treatment of tramadol were used in the carrageenan model of inflammatory pain/edema. In the first scheme, tramadol (1.25, 5, and 10 mg/kg) was administered systemically (i.p.) 10 min before carrageenan, and in the second scheme, tramadol (0.125 mg/paw) was coadministered locally (i.pl.) with carrageenan. To exclude systemic effects, the same dose of tramadol was administered to the contralateral paw. In the third scheme, the prophylactic treatment of systemically administered tramadol was modulated with magnesium sulfate (5 and 30 mg/kg), which was administered s.c. 5 min after tramadol. For magnesium, different doses were tested; the doses were chosen according to previous dose-dependent studies performed in our laboratory (Srebro et al., 2014a).

Two distinct schemes of therapeutic treatment of tramadol were used in carrageenan model of inflammatory pain/edema. In the first scheme, tramadol (1.25 mg/kg) was administered systemically (i.p.) 2 h after carrageenan, and in the second scheme, the therapeutic treatment of systemically administered tramadol was modulated with magnesium sulfate (5 and 30 mg/kg), which was administered s.c. 5 min after tramadol.

### Statistical Analysis

Data are expressed as mean differences in pressure d (g)/volume d (ml) ± standard errors of the mean (SEM) obtained in six rats. Statistical comparisons were made by two-way analysis of variance (ANOVA) with repeated measures, followed by Tukey’s HSD *post hoc* test. Student’s *t*-test was used for independent samples. *p* < 0.05 was considered as statistically significant.

## Results

### Prophylactic Effect of Systemic Tramadol on Inflammatory Pain and Edema in Rats

I.p. administration of tramadol (1.25, 2.5, or 10 mg/kg) before carrageenan-induced inflammation produced a statistically significant reduction of edema and hyperalgesia (*F* = 5.0; *df* = 3; *p* = 0.01) to mechanical stimuli. Repeated ANOVA revealed a statistically significant change of the analgesic (*F* = 4.38; *df* = 13.8; *p* = 0.000) and antiedematous effect (*F* = 58.64; *df* = 15.73; *p* = 0.000) with time. The maximal antihyperalgesic effect was about 68.8 ± 14–100% and developed during1 h after inflammation induction (Figure 1). The antihyperalgesic effect lasted up to 24 h. The maximal antiedematous effect was about 41.7 ± 12–100% and developed during 1 h after inflammation induction (Figure 2). The average differences in the paw withdrawal threshold and paw volume were decreased throughout the experiment in the different tramadol groups. However, with the exception of the some time points, tramadol did not produce a statistically significant dose-dependent antihyperalgesic and antiedematous effects. There were no significant differences in the baseline paw withdrawal threshold and paw volume between the groups tested (not shown).

**FIGURE 1:** The prophylactic effect of systemic tramadol on carrageenan -induced mechanical hyperalgesia. The abscissa presents the time after the injection of carrageenan. The ordinate presents the difference in pressures (g) applied to the plantar surface of the paw before and after injection of drugs. Significance: ^∗^*p* < 0.05 and ^∗∗^*p* < 0.01 by comparison with the curve for saline. Significance: ^+^*p* < 0.05 ^++^*p* < 0.01 between tramadol 2.5 and tramadol 1.25 or 10. Carr, carrageenan.

**FIGURE 2:** The prophylactic effect of systemic tramadol on carrageenan -induced inflammatory edema. The abscissa presents the time after the injection of carrageenan. The ordinate presents the difference in volume (ml) before and after injection of drugs. Significance: ^∗^*p* < 0.05 and ^∗∗^*p* < 0.01 by comparison with the curve for saline. Significance: ^+^*p* < 0.05 and ^++^*p* < 0.01 between tramadol 2.5 and tramadol 1.25 with tramadol 10. Carr, carrageenan.

### Therapeutic Effect of Systemic Tramadol on Inflammatory Pain and Edema in Rats

At the time when carrageenan-induced inflammation was maximally developed, i.p. administration of tramadol (1.25 mg/kg) produced a statistically significant reduction of the hyperalgesia to mechanical stimuli (*F* = 14.6; *df* = 1; *p* = 0.003) during the tested time (*F* = 4.86; *df* = 3; *p* = 0.007) (Figure 3). The maximal effect of about 51.8 ± 15% was observed at the 3 and 4 h time points. Under same conditions, tramadol significantly reduced the edema (*F* = 58; *df* = 1; *p* = 0.000) during the tested time (*F* = 8.06; *df* = 4; *p* = 0.003) (Figure 4). The antiedematous effect was 42.1 ± 6.9%, 49.4 ± 7.6%, 43.8 ± 8.8%, 51.4 ± 4.5%, and 58.8 ± 10.6% at the 3, 4, 5, 6, and 24 h time points, respectively. There were no significant differences in the baseline paw withdrawal threshold/paw volume between the groups tested (not shown).

**FIGURE 3:** The therapeutic effect of systemic tramadol on carrageenan – induced mechanical hyperalgesia. The abscissa presents the time after the injection of carrageenan. The ordinate presents the difference in pressures (g) applied to the plantar surface of the paw before and after injection of drugs. Significance: ^∗∗^*p* < 0.01 by comparison with the curve for saline. Carr, carrageenan.

**FIGURE 4:** The therapeutic effect of systemic tramadol on carrageenan – induced inflammatory edema. The abscissa presents the time after the injection of carrageenan. The ordinate presents the difference in volume (ml) before and after injection of drugs. Significance: ^∗∗^*p* < 0.01 by comparison with the curve for saline. Carr, carrageenan.

### Prophylactic Effect of Local Peripheral Tramadol on Inflammatory Pain/Edema in Rats

I.pl. administration of tramadol (0.125 mg/paw) with carrageenan produced a statistically significant reduction of the development of mechanical hyperalgesia from about 20 ± 4.4% to 70.3 ± 11.3% (*F* = 6.44; *df* = 1; *p* = 0.03) (Figure 5). This effect began at 2 h after administration and lasted up to 24 h, when it was maximally developed (*F* = 6.25; *df* = 3.4; *p* = 0.001). Also, at the local peripheral site tramadol produced a significant (*p* < 0.05) reduction of the development of edema from about 55.5 ± 11.2–100% (Figure 6). This effect began at 1 h after administration and lasted up to 24 h, and maximally developed at the 1 h after administration when completely abolished pain. The same dose of tramadol injected into the contralateral (non-inflamed) paw had no influence on carrageenan-induced hyperalgesia/edema (not shown).

**FIGURE 5:** The prophylactic effect of local peripheral tramadol on carrageenan – induced mechanical hyperalgesia. The abscissa presents the time after the injection of carrageenan. The ordinate presents the difference in pressures (g) applied to the plantar surface of the paw before and after injection of drugs. Significance: ^∗^*p* < 0.05 by comparison with the curve for saline. Carr, carrageenan.

**FIGURE 6:** The prophylactic effect of local peripheral tramadol on carrageenan -induced edema. The abscissa presents the time after the injection of carrageenan. The ordinate presents the difference in paw volume (ml) before and after injection of drugs. Significance: ^∗^*p* < 0.05 and ^∗∗^*p* < 0.01 by comparison with the curve for saline. Carr, carrageenan.

### Influence of Tramadol-Magnesium-Sulfate Administration on Mechanical Hyperalgesia/Edema

Tramadol (1.25 mg/kg, i.p.) was combined with different doses of magnesium sulfate (5 and 30 mg/kg, s.c.) and tested under both prophylactic and therapeutic protocols of use (Figures 7–10). Compared with saline, all groups treated with the tramadol-magnesium combination, or with tramadol or magnesium alone, produced a statistically significant analgesic/antiedematous effect in the carrageenan-induced inflammation test, which significantly changed in time. There were no statistically significant differences among the groups at baseline assessment of the paw withdrawal threshold/paw volume.

**FIGURE 7:** The prophylactic effect of tramadol (1.25 mg/kg) – magnesium sulfate (5 or 30 mg/kg) interaction on carrageenan – induced mechanical hyperalgesia. The abscissa presents the time after the injection of carrageenan. The ordinate presents the difference in pressures (g) applied to the plantar surface of the paw before and after injection of drugs. Significance: ^∗^*p* < 0.05 and ^∗∗^*p* < 0.01 by comparison with the curve for saline. Significance: between magnesium 30 + tramadol 1.25 and tramadol 1.25 (^+^*p* < 0.05 and ^++^*p* < 0.01). Carr, carrageenan; T 1.25, tramadol 1.25 mg/kg; MS 5, magnesium sulfate 5 mg/kg; MS 30, magnesium sulfate 30 mg/kg.

**FIGURE 8:** The prophylactic effect of tramadol (1.25 mg/kg) – magnesium sulfate (5 or 30 mg/kg) interaction on carrageenan – induced edema. The abscissa presents the time after the injection of carrageenan. The ordinate presents the difference in paw volume (ml) before and after injection of drugs. Significance: ^∗^*p* < 0.05 and ^∗∗^*p* < 0.01 by comparison with the curve for saline; ^+^*p* < 0.05 and ^++^*p* < 0.01 by comparison with the curve for tramadol 1.25. Carr, carrageenan; T 1.25, tramadol 1.25 mg/kg; MS 5, magnesium sulfate 5 mg/kg; MS 30, magnesium sulfate 30 mg/kg.

**FIGURE 9:** The therapeutic effect of tramadol (1.25 mg/kg) – magnesium sulfate (5 or 30 mg/kg) interaction on carrageenan- induced mechanical hyperalgesia. The abscissa presents the time after the injection of carrageenan. The ordinate presents the difference in pressures (g) applied to the plantar surface of the paw before and after injection of drugs. Significance: ^∗^*p* < 0.05 and ^∗∗^*p* < 0.01 by comparison with the curve for saline. Significance: ^+^*p* < 0.05 and ^++^*p* < 0.01 between tramadol 1.25 and magnesium 5 or 30 + tramadol 1.25. Carr, carrageenan, T 1.25, tramadol 1.25 mg/kg; MS 5, magnesium sulfate 5 mg/kg.

**FIGURE 10:** The therapeutic effect of tramadol (1.25 mg/kg) – magnesium sulfate (5 or 30 mg/kg) interaction on carrageenan – induced edema. The abscissa presents the time after the injection of carrageenan. The ordinate presents the difference in paw volume (ml) before and after injection of drugs. Significance: ^∗^*p* < 0.05 and ^∗∗^*p* < 0.01 by comparison with the curve for saline; ^++^*p* < 0.01 by comparison with the curve for tramadol 1.25. Carr, carrageenan; T 1.25, tramadol 1.25 mg/kg; MS 5, magnesium sulfate 5 mg/kg; MS 30, magnesium sulfate 30 mg/kg.

### Prophylactic Use of the Tramadol-Magnesium-Sulfate Combination in Rats With Inflammatory Pain and Edema

When magnesium sulfate at doses of 5 or 30 mg/kg were added to tramadol (1.25 mg/kg) before carrageenan-induced inflammation, the antihyperalgesic effect of tramadol was reduced by 50.1 and 39.5% at the 1 and 2 h time points, respectively (Figure 7). This effect was statistically significant (*F* = 6.05; *df* = 3; *p* = 0.004) only with the high dose of magnesium sulfate (30 mg/kg) (Figure 7). After this time point, magnesium sulfate at a dose of 30 mg/kg significantly (*F* = 8.14; *df* = 12.8; *p* = 0.000) prolonged the antihyperalgesic effect of tramadol at the 3, 5, and 6 h time points. Although magnesium at 30 mg/kg did not produce a statistically significant increase of the analgesic effect of tramadol, the average difference in the paw withdrawal threshold was decreased in comparison with other groups. The analgesic effects of the combination of tramadol and 30 mg/kg magnesium sulfate were 52.5 ± 11.6%, 20.8 ± 8.2%, and 22.7 ± 6.3% at the 3, 4, and 6 h time points, respectively. Tramadol alone at a dose of 1.25 mg/kg reduced carrageenan-induced mechanical hyperalgesia by about 100%, and by 56.3 ± 10.2% at the 1 and 2 h time points, respectively, magnesium at a dose of 5 mg/kg reduced mechanical hyperalgesia by about 65% at the 1 h time point, and by 53% at the 2 and 3 h time points, and magnesium at a dose of 30 mg/kg lowered the hyperalgesia by about 45% at the1 and 2 h time points.

When magnesium sulfate at doses of 5 or 30 mg/kg were added to tramadol (1.25 mg/kg) before carrageenan-induced inflammation, the antiedematous effect of tramadol was significantly increased at the 3, 4, 5, 6, and 24 h time points (Figure 8). Only in the 1 h time point magnesium sulfate at dose of 5 mg/kg abolished the antiedematous effect of tramadol. After this time point magnesium sulfate (5 mg/kg) significantly (*F* = 12.86; *df* = 3; *p* = 0.000) increased the antiedematous effect of tramadol during the time (*F* = 35.0; *df* = 4.16; *p* = 0.000). The antiedematous effects of the combination of tramadol and 5 mg/kg magnesium sulfate were 38.6 ± 6.2%, 34 ± 4.8%, 41.8 ± 4.8, 52.1 ± 2.5, and 75.5 ± 8.8% at the 3, 4, 5, 6, and 24 h time points (Figure 8). Magnesium sulfate at dose of 30 mg/kg significantly increased (*F* = 9.35; *df* = 3; *p* = 0.000) the antiedematous effect of tramadol during the time (*F* = 32.47; *df* = 4.36; *p* = 0.000) (Figure 8). The antiedematous effects of the combination of tramadol and 30 mg/kg magnesium sulfate were 41.4 ± 6.8%, 49.4 ± 4.6%, 41.0 ± 4.1%, and 71.6 ± 6.9% at the 3, 4, 6, and 24 h time points, respectively. Given alone, tramadol (1.25 mg/kg) or magnesium sulfate (5 or 30 mg/kg) reduced carrageenan-induced edema by about 14–20% and 20–40%, between the 3 and 6 h time points, respectively.

### Therapeutic Use of the Tramadol-Magnesium-Sulfate Combination in Rats With Inflammatory Pain/Edema

When magnesium was provided with tramadol (1.25 mg/kg) at the 2 h time point when the inflammatory pain was maximally developed, at doses of 5 or 30 mg/kg magnesium sulfate used in combination produced a statistically significant (*F* = 7.23; *df* = 3; *p* = 0.002 and *F* = 10; *df* = 3; *p* = 0.000, respectively) reduction in hyperalgesia to mechanical stimuli (Figure 9) at 3, 4, and 5 h time points. Only at dose of 30 mg/kg magnesium significantly (*F* = 3.81; *df* = 10.8; *p* = 0.000) prolonged the analgesic effect of tramadol (Figure 9). Both doses of magnesium sulfate (5 or 30 mg/kg) enhanced antihyperalgesic effect of tramadol for about 20% at the 4 and 5 h time points, respectively. The antihyperalgesic effect of the combination of tramadol and 30 mg/kg magnesium sulfate lasted 3 h and was 74.2 ± 6.7%, 70.5 ± 5.2%, and 49.0 ± 8.1% at the 3, 4, and 5 h time points, respectively (Figure 9). Tramadol alone reduced pain by about 25–51% at the 3 and 4 h time points, and by about 20% at the 5 and 6 h time points, and magnesium reduced pain by about 25–35% from the 3 to the 6 h time points. There were no statistically significant differences among the groups at baseline assessment of the paw withdrawal threshold.

Administration of tramadol (1.25 mg/kg) and magnesium sulfate (5 and 30 mg/kg) when the inflammatory edema was maximally developed resulted that magnesium sulfate at dose of 5 mg/kg abolished the antiedematous effect of tramadol (*F* = 15.53; *df* = 3; *p* = 0.000) and the dose of 30 mg/kg of magnesium sulfate significantly decreased (*F* = 23.0; *df* = 3; *p* = 0.000) the antiedematous effect of tramadol during the tested time (*F* = 23.05; *df* = 2.73; *p* = 0.000) (Figure 10). Given alone, tramadol (1.25 mg/kg) or magnesium sulfate (5 or 30 mg/kg) reduced carrageenan-induced edema by about 14–40%.

## Discussion

This study for the first time shows that: (i) tramadol systemically applied has both prophylactic and therapeutic analgesic effects in inflammatory pain and edema; (ii) magnesium sulfate enhances and prolongs the analgesic effect of tramadol in inflammatory pain; (iii) a better analgesic effect is produced by the combination of tramadol and magnesium sulfate at the dose at which magnesium alone has a weak analgesic effect, (iv) the combination of tramadol and magnesium sulfate is better for treatment than for prevention of inflammatory pain; and (v) magnesium sulfate enhances the antiedematous effect of tramadol in prevention of inflammatory edema; while reduced it effect in treatment of inflammatory edema.

These findings are important because they clarify the protocol at which dose and combination of tramadol and magnesium sulfate can be used to treat inflammatory pain and edema. Since inflammatory pain develops after trauma, surgery and rheumatic or arthritic diseases, this pain is the most commonly treated clinical pain. Our results are in agreement with other studies showing that both tramadol (Garlicki et al., 2006; Pecikoza et al., 2017) and magnesium sulfate (Srebro et al., 2014a, Vuckovic et al., 2015; Srebro et al., 2018a) have an analgesic effect in inflammation. Alexa et al. (2015) showed that magnesium enhanced the analgesic effect of tramadol in thermal nociceptive tests without inflammation or neuropathy. We used the carrageenan-induced mechanical inflammatory hyperalgesia test since this model has a high predictive value in studies of analgesics in inflammation, and because it mimics the time course of relief of postoperative pain and other different types of persistent injury.

In the current study, we showed that the combination of tramadol and magnesium sulfate (30 mg/kg b.w.) that corresponds to the average recommended daily dose in humans (250–350 mg; Srebro et al., 2017) produces an improved antihyperalgesic effect. When used as a sole analgesic for inflammatory pain, magnesium is very effective even in smaller doses (Srebro et al., 2014a), although the highest analgesic doses of magnesium do not disturb motor coordination (Vuckovic et al., 2015). During the inflammation, beside the pain, magnesium as a sole drug may be effective for reducing inflammatory edema (our unpublished results). Since both tramadol and magnesium are possible central nervous system depressants, it is important to note that the analgesic dose of tramadol (1.25 mg/kg) (Pecikoza et al., 2017) and magnesium sulfate (30 mg/kg) (Vuckovic et al., 2015) used in the present study do not alter motor coordination. Previously, we showed that the doses of magnesium sulfate used herein did not change the serum concentration of magnesium above the referent range (Srebro et al., 2018a), and they did not result in an increase in plasma magnesium concentration above the toxic 3 mM concentration (Felsby et al., 1996). Also, as hypomagnesaemia is associated with the onset of inflammation or can worsen it, we previously showed that our experimental rats had a normal basal blood magnesium concentration (Srebro et al., 2018a).

Magnesium sulfate at the dose of 30 mg/kg enhanced and prolonged tramadol’s effect in the carrageenan-induced mechanical hyperalgesia test, with an average increase of over 25% pain inhibition that was prolonged for 1 h in comparison to tramadol alone, especially when applied at the time when hyperalgesia was maximally developed. The increased effect produced at the time when inflammation was maximally developed, and when central sensitization occurred, as well as the absence of a local peripheral analgesic effect of magnesium in inflammatory pain (Srebro et al., 2014a) suggest that magnesium enhanced the effect of tramadol within a spinal mechanism. Magnesium chloride at a higher dose (150 mg/kg, i.p.) partially decreased the analgesic effect of tramadol in the hot-plate test at the first time point, but not in the tail flick test (Alexa et al., 2015). In agreement with this, in the present study, magnesium sulfate at the higher dose (30 mg/kg, s.c.) decreased the antihyperalgesic effect of tramadol by about 40–50% at the 1 and 2 h time points. A possible explanation for this is that magnesium, through the activation of transient receptor potential vanilloid type 1 (TRPV1) channels (Srebro et al., 2015, Srebro et al., 2016b), reduced the antihyperalgesic effect of tramadol that was effected through peripheral activation of the mu-opioid receptor and consequently, through mu-opioid receptor-specific inhibition of the TRPV1 channels via G i/o proteins and the cAMP/PKA pathway. Also, the analgesic effect of tramadol includes the direct activation of the intracellular nitric oxide/cyclic guanosine monophosphate pathway in primary nociceptive neurons (Lamana et al., 2017), while magnesium, by activating the same pathway in peripheral afferent neurons, could decrease the effect of tramadol (Srebro et al., 2015). According to our results, we suggest that in the primary afferent activation and peripheral sensitization (the first phase of carrageenan-induced hyperalgesiatest), magnesium reduced the analgesic effect of tramadol, whereas in the late phase of the test and central sensitization, magnesium enhanced the effect of tramadol.

In current study, we demonstrated that magnesium under same conditions increased analgesic and antiedematous effects of tramadol in prophylactic protocol of use, while in therapeutic protocol of use magnesium increased analgesic and decreased antiedematous effects of tramadol. This suggest that is: (i) better to give tramadol with magnesium in prophylactic protocol of use in inflammatory conditions, since that we have two targets, both pain and edema; and that (ii) the same or associated mechanism(s), at least in part, involved in the analgesic and antiedematous effect of tramadol and magnesium after preemptive administration. It is well known that in the carrageenan model of inflammation are increased release of cytokines and reactive oxygen species (Vazquez et al., 2015) and that magnesium sulfate decreases the production of tumor necrosis factor alpha (TNF-α) and interleukins 6 (IL6) in postoperative serum (Aryana et al., 2014).

In our study, both opioid and non-opioid mechanisms of action contributed to the antihyperalgesic effect of tramadol. It is well known that opioids via activation of mu-opioid receptors at central and peripheral sites (Hylden et al., 1991; Whiteside et al., 2005) and serotonin/noradrenaline reuptake inhibitors (Jones et al., 2006) can reduce carrageenan-induced hyperalgesia. Therefore, the analgesic action of tramadol is contributions in 40% via opioid mechanism (Raffa et al., 1992; Frink et al., 1996) and in 60% via activation of descending antinociceptive systems and suppression of amine reuptake (Raffa et al., 1992; Giusti et al., 1997). Activation of α2-adrenergic receptors has been shown to inhibit nociceptive transmission in the spinal cord through presynaptic activity, and to inhibit the release of excitatory neurotransmitters from primary afferent terminals and postsynaptic sites (Ossipov et al., 2010). An additional non-opioid mechanism of the analgesic effect of tramadol is the direct activation of the intracellular nitric oxide pathway in the primary signaling nociceptive neurons (Lamana et al., 2017).

There are many possible mechanisms for the analgesic effect of magnesium, such as: (1) Ca^++^ channel blocking, (2) decreasing the effects of acetylcholine on muscle receptors and increasing the threshold of axonal excitation (Dubé and Granry, 2003), (3) antagonism of NMDA receptors, (4) activation of transient receptor potential cation channel vanilloid type 1 (TRPV1), vanilloid type 4 (TRPV4), ancyrin type 1 (TRPA1) proteins (Srebro et al., 2016b), (5) NMDA-independent nitric oxide modulation of the antihyperalgesic effects of magnesium sulfate in inflammatory pain (Vuckovic et al., 2015; Srebro et al., 2014a,b, 2016a), (6) reducing inflammatory edema, and (7) an additional antiinflammatory mechanism (Aryana et al., 2014). A meta-analysis of randomized, controlled trials that included over 1,000 patients revealed that perioperative magnesium administration reduced both pain and opioid consumption (De Oliveira et al., 2013). Also, magnesium might be involved in the modulation of opioid receptors; the opioid-independent mechanism of the analgesic effect of magnesium is underscored (Murphy et al., 2013).

Additional information regarding the interaction with tramadol are that: (1) magnesium may have a permissive effect on catecholamine actions and that it can also inhibit norepinephrine release from nerve endings (Shimosawa et al., 2004), (2) that both drugs could affect the NO system, with magnesium increasing NO production (Srebro et al., 2014a) and tramadol directly activating the intracellular nitric oxide/cyclic guanosine monophosphate pathway in primary nociceptive neurons (Lamana et al., 2017), and (3) it is possible that magnesium potentiates the effect of tramadol in pain, since it has been shown that another NMDA antagonist increased the effect of tramadol in learning via activation of NO signaling pathway in brain (Jafari-Sabet et al., 2018). The potentiating effect of trace elements as adjuvant analgesics at different concentrations on an analgesic compound suggests that the analgesic effect is the consequence of the synergistic interaction between magnesium and tramadol.

This study has several limitations. Isobolographic analyses to verify type of interaction between tramadol and magnesium were not performed. The exact mechanisms through which the coadministration of magnesium enhanced the effect of tramadol have not been assessed. In addition, we did not perform pharmacokinetic research of tramadol. These findings have a potential impact on the results, and further research is required to translate these findings into clinical practice.

## Conclusion

The results obtained in the rat model of inflammatory pain and edema indicates that the systemic administration of tramadol with magnesium sulfate can prevent and treat somatic pain and edema during inflammation. Interaction of tramadol with magnesium is potent and effective. This is a safe combination for preemptive, and in particular for an emptive strategy to treat pain associated with inflammation. The best result is achieved when tramadol is combined with magnesium sulfate at a dose that is equivalent to the average human recommended daily dose and when the drugs are administered when inflammation is maximally developed. This combination presents an improvement to the current treatment of pain because the addition of an inexpensive dietary supplement such as magnesium helps reduce inflammatory pain and the dose of tramadol required to obtain analgesia.

## Author Contributions

DS and SV designed the experiment and analyzed the data. DS performed the experiments. DS wrote the main manuscript text. All authors revised the manuscript.

## Conflict of Interest Statement

The authors declare that the research was conducted in the absence of any commercial or financial relationships that could be construed as a potential conflict of interest.
